# Overexpression of 14-3-3*σ* Modulates Cholangiocarcinoma Cell Survival by PI3K/Akt Signaling

This article has been retracted.

**DOI:** 10.1155/2020/3740418

**Published:** 2020-06-22

**Authors:** Qiao Wu, Hua Fan, Ren Lang, Xianliang Li, Xingmao Zhang, Shaocheng Lv, Qiang He

**Affiliations:** Department of Hepatobiliary Surgery, Beijing Chao Yang Hospital, Capital Medical University, Beijing 100020, China

## Abstract

The protein 14-3-3*σ* is involved in numerous cellular processes through its ability to bind phosphorylated serine/threonine residues. It is a key regulator of the cell cycle involving in G2 arrest by p53. Deregulation of 14-3-3*σ* expression has been associated with a large variety of human cancers. However, its physiological function and therapeutic significance have rarely been investigated in cholangiocarcinoma. Using immunohistochemistry (IHC), we evaluated 14-3-3*σ* expression in 65 human extrahepatic cholangiocarcinomas. As a result, we found that 14-3-3*σ* is expressed in the tissue of 56 patients (86.2%), and its expression is positively correlated with tumor size, lymph node metastasis, and tumor stage. We also explored the significance of 14-3-3*σ* and found that 14-3-3*σ* exerts cell type-dependent effects on cell proliferation through PI3K/Akt signaling in both *in vitro* and *in vivo* xenograft models. These results suggest that 14-3-3*σ* assumes a constitutive role in tumorigenesis rather than acting as a cell cycle regulator in cholangiocarcinoma, which makes 14-3-3*σ* a new potential target for therapeutic intervention.

## 1. Introduction

Cholangiocarcinoma (CCA) is a rare malignancy with devastating outcomes. Tumors can arise from the lining of the bile duct epithelium anywhere [1, 2]. Depending on their anatomical location, CCAs are categorized as intrahepatic or extrahepatic CCA; the individual categories differ in terms of biological behavior, clinical presentation, and management [3]. While numerous risk factors for CCA are known, the pathogenesis of this disease is still obscure [1, 4–6]. In clinical practice, extrahepatic CCAs are usually asymptomatic at early stages and are often diagnosed at an advanced stage of the disease. For the last four decades, the worldwide incidence of CCA progressively increased [7]. Surgical excision is considered to be the most effective therapeutic route for CCA; however, the 5-year survival rate remains around 20–30% [8, 9]. Therefore, it is paramount to identify novel tumor markers for this disease that will allow early detection, as well as new potential targets for therapeutic intervention [10].

14-3-3 proteins are highly conserved. In mammals, seven distinct isoforms are known (*β*, *σ*, *γ*, *θ*, *δ*, *ε*, and *η*). The 14-3-3 proteins are crucial regulators of intracellular signaling pathways. The physiological function of these proteins is still unclear. However, through binding to diverse target proteins, 14-3-3 proteins appear to be involved in a wide variety of cellular processes, such as cell proliferation, cell cycle progression, apoptosis, signal transduction, and malignant transformation [11, 12].

14-3-3*σ*, also called stratifin, belongs to the 14-3-3 family; it was first identified as an epithelial-specific marker (HME1). This protein is mostly expressed in human epithelial cells and is involved in various processes such as signal transduction and growth regulation. Accumulating data indicate that 14-3-3*σ* can bind to other important proteins associated with tumor initiation and development through its ligand-binding domain. Silencing of 14-3-3*σ* due to hypermethylation of the CpG island has been observed in breast cancer [13–15], lung cancer [16], ovarian cancer [17], hepatocellular carcinoma [18], and certain squamous cell carcinomas [19]. In contrast, 14-3-3*σ* appears to be upregulated in gastric cancer [20], colon carcinoma [21], pancreatic cancers [22, 23], and head and neck squamous cell carcinoma [24].

To date, there is no data on the role of the 14-3-3*σ* on CCA initiation and development. Here, we assess the expression of 14-3-3*σ* in CCA as well as its potential role as a regulator of the essential signaling proteins involved in relaying the inputs from multiple upstream survival pathways in CCA.

## 2. Materials and Methods

### 2.1. Tumor Samples

Sixty-five surgically resected samples were collected from patients diagnosed with extrahepatic cholangiocarcinoma according to radiologic findings with no preceding therapy at the Department of Hepatobiliary Surgery, Beijing Chao Yang Hospital, Capital Medical University, from January 2010 to September 2013. Clinicopathological data including age, sex, tumor size, pathologic differentiation, lymphatic permeation, and tumor stage are reported in Table 1. Depending on their degree of papillary or tubular formation, tumors were distributed into 3 groups (30 well-differentiated, 29 moderately differentiated, and 6 poorly differentiated). If more than one type was observed, the tumor was classified according to the most prominent type. The tumor histologic stage was defined from stage I to stage IVB based on histologic examination according to the pTNM classification issued by the International Union Against Cancer. The prognosis was collected by reviewing patient case records. Specimens were fixed with 10% formalin and embedded in paraffin wax.

### 2.2. Tissue Preparation and Antibodies

The histologic sections of extrahepatic cholangiocarcinoma fixed in paraffin were rehydrated and dewaxed. Antigen retrieval was carried out after endogenous peroxidase activity has been blocked through incubation with 3% hydrogen peroxide in absolute methanol for 10 minutes. The histologic sections were incubated for 1 h at 37°C with the primary antibody directed toward 14-3-3*σ* isoform (Santa Cruz, CA); the primary antibody was diluted to 1 : 200 ratio. The slides were then incubated for 50 minutes at ambient temperature with a secondary antibody (Dako). The histologic sections were visualized with 3,3-diaminobenzidine (DAB) and counterstained with Mayer's hematoxylin. The methods we used in this part are the same as what we did previously [25].

### 2.3. Scoring of Immunoreactivity

The intensity of IHC staining in tumor cells was scored independently by two pathologists that were blinded to the clinicopathological data following the semiquantitative IRS (immunoreactive score) scale. The final score was defined as the average from the two referees. 14-3-3*σ* staining intensity (14-3-3*σ*-SI), percentage of 14-3-3*σ*-positive tumor cells (14-3-3*σ*-PP), and a resulting 14-3-3*σ* immunoreactivity score (14-3-3*σ*-IRS) were all determined following a slightly modified version of the protocol published elsewhere [26]. Briefly, the immunoreactivity score (14-3-3*σ*-IRS: negative 0, weak 1–3, moderate 4–6, and strong 8–12) was obtained by multiplying the values for 14-3-3*σ* staining intensity (14-3-3*σ*-SI: 0, no staining; 1, weak staining; 2, moderate staining; and 3, strong staining) and the values for percentage of 14-3-3*σ*-positive tumor cells (14-3-3*σ*-PP: score 1, 0-10%; score 2, 11-25%; score 3, 26-50%; and score 4, >51%).

### 2.4. Cell Lines and Cell Culture

The TFK-1 cell line was obtained from the Department of Biochemistry (Chinese Academy of Medical Sciences and Peking Union Medical College, China) and grown in Dulbecco's modified Eagle's medium (DMEM, Hyclone, Thermo Fisher Scientific Inc., Waltham, MA) supplemented with 10% fetal bovine serum (FBS, Hyclone), 100 U penicillin, and 100 mg/mL streptomycin. All cells were grown at 37°C with 5% CO_2_ in a humidified incubator. The human CCA cell line TFK-1 underwent lentiviral transduction to stably silence 14-3-3*σ*.

### 2.5. Transient Transfection

A specific 14-3-3*σ* small interfering RNA (siRNA) was designed according to the cDNA sequence of 14-3-3*σ* (sequence: 5′-UGAAGAUGAAGGGUGACUATT-3′). The negative control is a scrambled nontarget siRNA. The siRNAs were synthesized by Invitrogen Company (Shanghai, China). Lipofectamine 2000 (Invitrogen) was used for siRNA transfection in TFK-1 cells following the manufacturer's instructions. 24 h after transfection, TFK-1 cells were used in CCK8, flow cytometry assay, and Transwell migration assays. The expression level of 14-3-3*σ* was monitored by western blot.

### 2.6. Western Blot Analysis

The rabbit anti-14-3-3*σ* was from Santa Cruz (Santa Cruz, CA). Antibodies against p-Bad (cat # 4366S), p21 (cat # 2946S), cyclin D1 (cat # 2926P), p-GSK-3*α*/*β* (cat # 9331S), PTEN (cat # 9559S), p-PI3K (cat # 4228S), p-AKT (cat # 4060S), p27 (cat # 2559P), Bax (cat # 2772S), Bad (cat # 9292S), and *β*-actin (cat # 4970S) were purchased from Cell Signaling Technologies (Danvers, MA). Cells were harvested though trypsinization followed by centrifugation. Pelleted cells were lysed in lysis buffer supplemented with protease inhibitors and processed for western blotting.

### 2.7. Cell Proliferation Assay

Cell proliferation was measured with the cell count kit (CCK-8, Domino, Shanghai, China). In short, cells were seeded in 96-well plates at 5 × 10^3^ cells/well and transfected with 14-3-3*σ* siRNA or a negative control. 48 hours after transfection, the CCK-8 assay was performed. Transfected cells were incubated with culture medium containing the CCK-8 reagent for 4 hours; the absorbance was read at 450 nm using a microplate enzyme-linked immunosorbent assay reader (Labsystems Dragon, Wellscan).

### 2.8. Flow Cytometry Assay of Cell Apoptosis

Cells were harvested by trypsinization, collected by centrifugation, and washed once with phosphate-buffered saline (PBS). Cells were then fixed at 4°C in 1 mL of 75% ethanol. Cells were washed once more with PBS before a 30 min incubation at room temperature in 1 mL PBS supplemented with 30 *μ*g/mL propidium iodide and 0.25 mg/mL RNase A. Cells were analyzed for DNA content by flow cytometry using FACS (fluorescence-activated cell sorter) Cytomics FC 500 (Beckman). The data were treated with Multicycle AV for Windows (Beckman). Apoptosis was induced by 10 *μ*g/mL of gemcitabine.

### 2.9. *In Vitro* Migration Assays

The cell migratory abilities were determined by Transwell assays. Cell culture inserts with 8 *μ*m microporous filters without extracellular matrix coating (Becton Dickinson Labware, Bedford, MA) were seeded with 5.0 × 10^4^ TFK-1 cells in 200 *μ*L serum-free DMEM. The bottom chambers were loaded with 500 mL DMEM containing 10% FBS. Following a 24 h incubation period, noninvading cells were gently removed with a cotton swab. Migrating cells located on the lower surface of the chamber were stained with the Diff-Quick Staining Set (Dade) and counted under a microscope.

### 2.10. Stable Transduction

The 14-3-3*σ* miRNA-interfering (14-3-3*σ*-miR) and normal control (control-miR) cell lines were generated through lentiviral transduction. 14-3-3*σ*-miR was transduced with lentivirus containing an oligo antisense sequence of 14-3-3*σ*. Lentiviral particles were obtained by cotransfection of Packaging Mix with Opti-MEM and Lipofectamine 2000 (Life Technologies). The supernatants containing the virus were concentrated using ultracentrifugation at 50,000 g for 2 h. TFK-1 cells grown in 12-well plates were infected in the presence of 8 *μ*g/mL Polybrene (Sigma-Aldrich). The transduced cells were identified using blasticidin (0.5 mg/mL-10 mg/mL).

### 2.11. Xenograft Studies

BALB/c nu/nu female mice were raised in an SPF room. TFK-1 cells were injected subcutaneously into the right axillary area of the 4-week-old mice. Mice were sacrificed 30 days later, and the tumor size and weight were measured.

### 2.12. Statistics

Statistical analyses were made with the SPSS 13.0 software (SPSS, Chicago, IL). Continuous data were presented as the mean ± standard deviation (SD) calculated from at least 3 individual duplicated experiments. Statistical significance was calculated by Student's *t*-test. A value of *P* < 0.05 was considered statistically significant.

## 3. Results

### 3.1. Immunohistochemistry

In order to evaluate the expression of 14-3-3*σ* in extrahepatic cholangiocarcinoma, we first examined the presence of the protein in tissue samples from 65 patients by immunochemistry (patient details are summarized in Table 1). Positive cells showed an intense staining in the cytoplasm (see Figure 1 for cases typically evaluated as positive or negative). 56 cases were evaluated as 14-3-3*σ*-positive (86.2%) against 9 evaluated as negative (13.8%). 19 cases (out of 56: 35.8%) had 14-3-3*σ*-positive cancer tissue adjacent to morphologically normal glands. Immunoreactivity toward 14-3-3*σ* is significantly different between extrahepatic cholangiocarcinoma tissue and adjacent normal bile ducts.

### 3.2. Correlation between 14-3-3*σ* Expression and Clinicopathological Parameters

Since 14-3-3*σ* seems to be expressed in 86% of extrahepatic cholangiocarcinoma, we explored the connection between 14-3-3*σ* and clinicopathological factors. As can be seen in Table 2, expression of 14-3-3*σ* significantly correlates with tumor size (*P* = 0.02), lymph node metastasis (*P* = 0.027), and tumor stage (*P* = 0.01).

There was, however, no significant relationship between 14-3-3*σ* expression and patient sex, age, pathologic differentiation, and serum tumor markers (CEA, CA-242, or CA19-9).

### 3.3. Correlation between 14-3-3*σ* Expression and Clinical Outcome

The overall survival curve of 65 extrahepatic cholangiocarcinomas following the Kaplan-Meier method is shown in Figure 2. The 1-, 3-, and 5-year survival rates were 100%, 77.8%, and 44.4% for the 14-3-3*σ*-negative group compared to 73.2%, 21.4%, and 1.8% for the 14-3-3*σ*-positive group. 14-3-3*σ*-positive cases showed significantly worse prognosis than 14-3-3*σ*-negative cases (*P* = 0.014).

The univariate analysis by Cox (Table 3) reveals that tumor size (*P* = 0.02), lymph node metastasis (*P* = 0.027), tumor stage (*P* = 0.001), and 14-3-3*σ* level (*P* = 0.034) are significantly correlated with a worse prognosis for overall survival in 65 extrahepatic cholangiocarcinoma patients. Multivariate analysis (Table 3) shows that the tumor stage (*P* = 0.041) and 14-3-3*σ* level (*P* = 0.033) are independent prognostic factors with relative risks of 2.29 and 9.28, respectively.

### 3.4. Silencing of 14-3-3*σ* Inhibits Cell Growth and Reduces S Phase Cell Ratio

Since 14-3-3*σ* expression is associated with aggressive tumor features, we examined next the influence of 14-3-3*σ* on the proliferative potential in CCA cells. TFK-1 cell lines were engineered to express either a siRNA targeting 14-3-3*σ* expression or a scrambled nontarget siRNA. As detected by western blot (Figure 3(a)), siRNAs targeting 14-3-3*σ* treatment caused severe 14-3-3*σ* suppression (Figure 3(b)). As can be seen in Figure 3(c), suppression of 14-3-3*σ* expression for 4 days reduced the proliferation rate of TFK-1 cells.

To determine the origin of this reduced cell proliferation rate, the cell cycle distribution of these cell lines was analyzed by flow cytometry. Following the suppression of 14-3-3*σ* expression, the fraction of cells in G1 phase increased (Figure 3(e)) while the proportion of cells in S phase decreased (Figure 3(d)), suggesting that 14-3-3*σ* suppression can induce slight G1 arrest (Supplementary Fig 1).

### 3.5. Effects of 14-3-3*σ* Suppression in TFK-1 Cells on Gemcitabine-Induced Apoptosis

To determine whether silencing of 14-3-3*σ* would make CCA cells more sensitive to gemcitabine, we quantified cell apoptosis using flow cytometry. In response to 1 *μ*M gemcitabine, cells transfected with 14-3-3*σ* siRNA exhibited increased apoptosis compared to cells transfected with scrambled siRNA (Figures 4(a) and 4(b)).

### 3.6. 14-3-3*σ* Is Not Required for the Regulation of Metastatic Potential in TFK-1 Cells

The impact of 14-3-3*σ* on metastatic potential was assessed by Transwell assays. For TFK-1 cells, no significant difference in motility could be measured between cells transfected with 14-3-3*σ* siRNA and cell transfected with the scrambled siRNA (data not shown).

### 3.7. 14-3-3*σ* Regulates PI3K/Akt Pathway and p53 in TFK-1 Cells

Since knocking down 14-3-3*σ* in TFK-1 cells modified their proliferative and survival properties, we assessed the expression levels of related proteins by western blot in order to identify the molecular network underlying these observations (Figure 5).

Silencing of 14-3-3*σ* seems to be associated with a downregulation of p-Akt but does not lead to any significant change in the levels of total Akt and its upregulation by p-PI3K. Cyclin D1 is downregulated, whereas p53, p27, and p21 are upregulated. Proapoptotic proteins (Bim and Bax) are dramatically upregulated. On the other hand, the antiapoptotic marker p-Bad is not significantly altered in response to 14-3-3*σ* suppression. Interestingly, the invasion suppressor E-cadherin does not seem to be significantly affected by downregulation of 14-3-3*σ* in TFK-1 cells.

### 3.8. Silencing of 14-3-3*σ* Inhibits Tumor Growth in BALB/C Nude Mice

To further investigate whether silencing of 14-3-3*σ* suppresses CCA tumor growth *in vivo*, stably transduced TFK-1 CCA cell lines were injected into the subaxillary regions of BALB/c nude mice (*n* = 8 in each group) (Supplementary Fig 2). The efficiency of stable transduction with lentivirus to extrahepatic cholangiocarcinoma cell line TFK-1 is about 78%-90% (Supplementary Fig 3). Tumor volume and weight were monitored in order to assess the proliferation speed of each group. Mice injected with 14-3-3*σ*-miR cells show significantly smaller tumor volume and weight compared to mice injected with control-miR cells (Figure 6). These observations suggest that silencing of 14-3-3*σ in vivo* can suppress CCA tumor growth.

Taken together, our results suggest that (i) 14-3-3*σ* is associated with a higher cell proliferation rate and a higher proportion of cells in S phase, (ii) 14-3-3*σ* plays a role in the chemoresistance of CCA toward gemcitabine, and (iii) 14-3-3*σ* may not be required for the regulation of the metastatic potential of CCA.

## 4. Discussion

14-3-3*σ* was first identified as a mammary epithelium marker. Only later was 14-3-3*σ* found to play a major role in the regulation of cell cycle checkpoints. In response to DNA damage, 14-3-3*σ* expressions are induced under the control of p53. Expression of 14-3-3*σ* leads to the sequestration of cyclin B1 to the cytoplasm, precluding it from entering the nucleus, consequently preventing the initiation of mitosis [13, 27]. Therefore, 14-3-3*σ* appears to act as a suppressor of cell cycle progression and is associated with cancer.

However, the role of 14-3-3*σ* as a tumor suppressor is questionable as 14-3-3*σ* can also be upregulated in some cancers. Indeed, in this study, we observe overexpression of 14-3-3*σ* in the tissue of 56 out of 65 CCA patients. We could also show that 14-3-3*σ* is related to CCA progression since overexpression of 14-3-3*σ* expression is an independent prognostic factor for CCA, which suggests that 14-3-3*σ* harbors a role in tumorigenesis and/or progression of CCA.

Based on this observation, we propose that 14-3-3*σ* stimulates CCA progression. In order to identify the molecular mechanisms at hand, we silenced the expression of 14-3-3*σ* in human CCA cell lines by transient and stable transfection. Using this experimental setup *in vitro* and in *in vivo* xenograft models, we could show that CCA cell growth and apoptosis are influenced by 14-3-3*σ*. Upregulation of 14-3-3*σ* leads to increased proliferation as well as resistance to apoptosis. These results indicate that 14-3-3*σ* shows an oncogenic potential as its expression is correlated with the expression of proteins involved in cancer initiation and progression. 14-3-3*σ* suppression seems to lead to G1 cell cycle arrest, increased gemcitabine-induced apoptosis, and reduced cell proliferation.

Next, we focused on the role of 14-3-3*σ* and its potential interplay with other key payers of cell cycle regulation as well as cell proliferation and invasion. We found that 14-3-3*σ* affects the PI3K/Akt pathways, by which dysregulation can lead to human cancers [28, 29]. The PI3K/Akt signaling pathways are known to be activated in CCA, regulating tumor growth and metastasis. Our western blot results revealed that downregulation of 14-3-3*σ* correlates with the downregulation of p-Akt but does not affect the levels of total Akt and its upregulation by p-PI3K. These observations suggest that 14-3-3*σ* could interfere with the phosphorylation of Akt and could maintain the proliferative abilities of the cell by activating the PI3K/Akt signaling cascade.

In addition to the PI3K/Akt pathway, 14-3-3*σ* appears to regulate other molecules in the p53 network. In response to 14-3-3*σ* suppression, p21, p27, and p53 were upregulated, leading to cell cycle arrest. Meanwhile, cyclin D1, a protein involved in the G1/S transition, was downregulated (Figure 7).

CCA exhibits substantial resistance to chemotherapies, targeted agents, and radiotherapy. Currently, gemcitabine appears to be a valid therapeutic option for CCA patients [30, 31]. Our results show that 14-3-3*σ* knockdown enhances sensitivity toward gemcitabine in CCA cells and leads to significant cell apoptosis. We also observed that proapoptotic molecules (Bim and Bax) were dramatically upregulated following 14-3-3*σ* knockdown.

14-3-3*σ* has been proposed to be involved in metastasis and cancer invasion; increased 14-3-3*σ* expression appears to significantly correlate with large tumor size and higher invasion in some cancers [19, 32]. However, we did not find a significant correlation between 14-3-3*σ* expression and metastatic potential in CCA cells, similarly to what was observed in T3M4 cells [33].

In summary, we provided new evidence exploring the functional roles of 14-3-3*σ* protein in bile duct tumorigenesis. We anticipate that the interaction between 14-3-3*σ* and upstream factors of the PI3K/Akt pathway and p53 network could raise consideration for 14-3-3*σ* inhibitors as a new avenue to treat CCA.

## Figures and Tables

**Figure 1:** Immunoreactivity of 14-3-3*σ* in extrahepatic cholangiocarcinoma specimens. Typical cases evaluated as negative (a) or positive (b) are shown.

**Figure 2:** Overall survival curves of 65 extrahepatic cholangiocarcinomas according to 14-3-3*σ* expression were generated using the Kaplan-Meier method. The statistical significance of differences in the survival analyses was calculated using the log-rank test. Significance was set as *P* < 0.014.

**Figure 3:** 14-3-3*σ* suppression inhibits cell growth, reduces the S phase cell ratio, and stimulates apoptosis in vitro. (a) Western blot for 14-3-3*σ* proteins for transduction. (b) Average ratio of normalized 14-3-3*σ* expression. ^∗^*P* < 0.05. (c) Relative proliferation at 1, 2, 3, and 4 d. ^∗^*P* < 0.05. (d) Relative number of cells in S phase, based on flow cytometry assay. (e) Relative number of cells in G1 phase, based on flow cytometry assay.

**Figure 4:** 14-3-3*σ* silencing leads to higher apoptosis rate. (a) Flow cytometry assay for apoptosis. (b) Relative rates of apoptosis, based on flow cytometry assay. ^∗^*P* < 0.05.

**Figure 5:** Western blotting for molecules critical for cell proliferation and apoptosis.

**Figure 6:** Silencing of 14-3-3*σ* inhibits tumor growth in nude mice. (a) Volume of tumors in each group, ^∗^*P* < 0.05. (b) Weight of tumors in each group. ^∗^*P* < 0.05.

**Figure 7:** 14-3-3*σ* may generate an increase in cell proliferation, an increase in the proportion of cells in S phase, and a contribution to the chemoresistance of CCA toward gemcitabine.

**Table 1:** Clinical and histopathological characteristics of 65 extrahepatic cholangiocarcinomas.

Characteristics	Value	No. of patients (%)
Gender (%)	Male	37 (56.9)
	Female	28 (43.1)
Age (%)	≥65 years	22 (33.8)
	<65 years	43 (66.2)
Tumor size (%)	>2.5 cm	35 (53.8)
	≤2.5 cm	30 (46.2)
Pathologic differentiation (%)	Well	30 (46.2)
	Moderate	29 (44.6)
	Poor	6 (9.2)
Lymphatic permeation (%)	No	27 (41.5)
	Yes	38 (58.5)
Tumor stage (%)	I+II	25 (38.5)
	III+IV	40 (61.5)
14-3-3*σ* level (%)	Negative	9 (13.8)
	Positive	56 (86.2)

**Table 2:** Clinical and histopathological characteristics according to 14-3-3*σ* status in 65 extrahepatic cholangiocarcinomas.

	14-3-3*σ* expression			*P* value
	Total (*n* = 65)	Negative (*n* = 9)	Positive (*n* = 56)	
Gender (%)				
Male	37 (56.9)	5 (55.6)	32 (57.1)	NS
Female	28 (43.1)	4 (34.4)	24 (42.9)	
Age (%)				
≥65 years	22 (33.8)	4 (34.4)	18 (32.1)	NS
<65 years	43 (66.2)	5 (55.6)	38 (67.9)	
Tumor size (%)				
>2.5 cm	45 (69.2)	3 (33.3)	42 (75.0)	0.020
≤2.5 cm	20 (30.8)	6 (66.7)	14 (25.0)	
Pathologic differentiation (%)				
Well	30 (46.2)	2 (22.2)	28 (50.0)	NS
Moderate	29 (44.6)	4 (44.4)	25 (44.6)	
Poor	6 (9.2)	3 (33.4)	3 (5.4)	
Lymphatic permeation (%)				
No	27 (41.5)	7 (77.8)	20 (35.7)	0.027
Yes	38 (58.5)	2 (22.2)	36 (64.3)	
Tumor stage (%)				
I+II	25 (38.5)	8 (66.7)	17 (32.1)	0.001
III+IV	40 (61.5)	1 (33.3)	39 (67.9)	

**Table 3:** Univariate and multivariate analyses of overall survival in 65 extrahepatic cholangiocarcinomas.

	Univariate	Multivariate	
	*P* value	*P* value	Relative risk (95% CI)
Gender	0.602		
Age	0.473		
Tumor size	0.020	0.173	2.51 (0.818–8.103)
Pathologic differentiation^1^	0.074		
Lymphatic permeation^1^	0.027	0.059	5.77 (0.449–11.017)
Tumor stage^1^	0.001	0.041	2.29 (1.152–12.845)
14-3-3*σ* level^1^	0.034	0.033	9.28 (2.416–19.577)

^1^Data were considered significant by univariate analyses and examined by multivariate analyses.

## Data Availability

The data used to support the findings of this study are available from the corresponding author upon request.

## Supplementary Materials

Supplementary Materials Supplementary Fig 1: 14-3-3*σ* suppression reduces the S phase cell ratio and induces slight G1 arrest in vitro. ^∗^*P* < 0.05. Supplementary Fig 2: silencing of 14-3-3*σ* (Group B) suppresses CCA tumor growth in BALB/c nude mice compared with control (Group A). Gross appearance of tumors from BALB/c nude mice in two groups. ^∗^*P* < 0.05. Supplementary Fig 3: the efficiency of stable transduction with lentivirus to extrahepatic cholangiocarcinoma cell line TFK-1 is about 78%-90%.
